The article "Traditional Chinese Medicine Moxibustion in the Treatment of Infantile Diarrhea" was retracted in 2023. Reasons: signs of a paper mill; compromised peer review; unreliable results or conclusions.

# Traditional Chinese Medicine Moxibustion in the Treatment of Infantile Diarrhea

**DOI:** 10.1155/2022/9749606

**Published:** 2022-06-30

**Authors:** Ziming Li

**Affiliations:** Graduate School of Tianjin University of Traditional Chinese Medicine, No.10 Poyang Lake Road, Tuanbo Xincheng West District, Jinghai District, Tianjin, China

## Abstract

The main contribution of this research paper is to summarize the results of Meta-analysis of moxibustion in the treatment of infantile diarrhea which is one the common disease and requires considerable attention from the research community and funding organizations. In order to verify that the proposed scheme has merits, a comprehensive searching methodology was adopted by considering various databases such as China Biomedical Literature Database (CBM), China National Knowledge Network Infrastructure (CNKI), Wanfang Database, Pub Med Database, Google Academic, and Cochrane Library. It is important to note that a powerful computer has been utilized to carry out this searching. Finally, only those literature contents are selected which meet the inclusion criteria. Likewise, exclusion criteria was used to exclude irrelevant contents of the literature. RevMan 5.3 was used to analyze the collected data and after reading the titles and abstracts, 29 well-designed studies were selected. Through searching the full text, reading literature, and quality evaluation, 17 papers were finally included. Response rates were reported in all 17 studies, and subgroup analysis was performed based on whether or not other therapies were combined. 7 studies compared the effectiveness of simple moxibustion and conventional therapy in the treatment of infantile diarrhea, and the results showed statistically significant differences [OR = 4.01, 95% CI (2.03, 7.84), *P* < 0.0001]; 10 studies compared the effectiveness of moxibustion combined with other therapies and conventional therapies in the treatment of diarrhea in children, and the results showed that the difference had general meaning [OR = 4.45, 95% CI (2.83, 7.10), *P* < 0.00001]. The funnel plot (in Figure) showed that the distribution of included studies was asymmetrical on both sides of the baseline, which could be considered as publication bias. Traditional Chinese medicine moxibustion could effectively relieve the symptoms of infantile diarrhea, and the effect was significant.

## 1. Introduction

Diarrhea is a digestive tract syndrome caused by multiple pathogens and factors. Likewise, it is fairly common, and it affects almost everyone at least once a year. Your face will be loose and runny if you have diarrhea. The cause is usually unclear, and it clears up on its own within a few days. Bacteria can lead to diarrhea. Diarrhea might cause dehydration, which is a serious adverse effect. Its main symptoms include excessive secretion and absorption disorder of intestinal mucosa, excessive intestinal peristalsis, change of normal intestinal habits, thinness of feces, and abnormal components [1]. Infantile diarrhea is a clinical syndrome caused by multiple pathogens and factors, which is characterized by the increased number of stools and changes in the characteristics of stools [2]. Infantile diarrhea in children is common in infants and young children, with a high incidence of disease. The main cause is the incomplete development of physical function in children, excessive diet, and improper feeding, resulting in the weakness of the spleen and stomach in children, resulting in a significant decline in digestive function. Because the food was not digested, the child showed increased stool frequency, abdominal distension, diarrhea, and loss of appetite [3]. When children maintain diarrhea for a long time, it will cause indigestion and various nutrition-related diseases, which will affect the growth of children [4]. Apart from it, a prolonged diarrhea may cause serious consequences and may severely effects the health status of the children. A large number of moxibustion treatments and medical cases are recorded in ancient books of Chinese medicine. Traditional Chinese medicine masters in the past dynasties all have their unique views on moxibustion, and there are a large number of related medical cases about the use of moxibustion for diarrhea [5]. Moxibustion treatment for infantile diarrhea in Traditional Chinese medicine has proven efficacy, is easy to use, safe, and painless and is well accepted by children and their families [6].

The article "Traditional Chinese Medicine Moxibustion in the Treatment of Infantile Diarrhea" was retracted in 2023. Reasons: signs of a paper mill; compromised peer review; unreliable results or conclusions.

In this paper, we have conducted a Meta-analysis of the existing Traditional Chinese medicine moxibustion, especially in the treatment process of infantile diarrhea. As diarrhea is assumed as the most common and crucial disease for human beings in general and children in particular. Therefore, we are interested in finding a reliable and efficient treatment plan for the diarrhea disease, especially children.

The rest of the paper is organized as follows.

In Section 2, i.e., Materials and Methods, we have described in detail how a group of patients or individuals are divided into various groups and the criteria that is used for the separation of the patients into groups. In addition, why some patients are not allowed or excluded from the experimental study is described. What we have achieved through these experiments are presented in the graphical format in the Results section i.e., Section 3. In addition, a detailed discussion of those results is also provided in Section 4. Finally, conclusion remarks are given at the end in Section 5.

## 2. Materials and Methods

### 2.1. Literature Inclusion and Exclusion Criteria

The inclusion and exclusion criteria were as follows:

 
*Inclusion Criteria*. ① In the literature, the experimental group was moxibustion therapy or moxibustion combined with other therapies whereas the control group was other therapies except for moxibustion therapy; ② all publicly published randomized controlled trials or semirandomized controlled trials of moxibustion in the treatment of pediatric diarrhea, whether or not using a blind method; ③ the age, gender, and origin of the children were not limited, and diarrhea met all the diagnostic criteria of pediatric diarrhea at home and abroad.
 
*Exclusion Criteria*. ① The data were incomplete or there are obvious statistical errors; ② the paper was repeatedly published or the full text was not available; ③ pathological reports, cases, reviews, and so on.

### 2.2. Literature Retrieval Method

Retrieve literature by database retrieval and keyword retrieval:

1. *Retrieve Database*. In this study, the relevant original pieces of literature published in Chinese databases were systematically searched, including Pub Med, Wanfang, CNKI, CBM, Google Academic, and Cochrane Library. The retrieval time was from the establishment of the database to November 2020. These databases were searched through a dedicated and preferably efficient computer system which is programmed such that the concerned exclusion and inclusion criteria are matched or rules for these criteria are followed.
2. *Retrieve Key Words*. Using the method of “subject words + free words,” the Chinese retrieval key words included: “infantile diarrhea,” “Traditional Chinese medicine moxibustion,” and “random.” The key word is an interesting feature, especially for the searching of databases or other records in the online repositories.

### 2.3. Literature Quality Evaluation and Literature Extraction

Methodological quality was evaluated according to the modified Jadad scale, which included random method, allocation concealment, blind check-out, and lost followup. The Jadad scale, often known as Jadad scoring or the Oxford quality score system, is a mechanism for evaluating a clinical trial's methodological quality independently. It was named after Colombian physician Alex Jadad, who established a technique for assigning a score of zero to five to such studies in 1996 (rigorous). The total score of the evaluation scale was 7 points, with 1–3 points representing low quality research and 4–7 points representing high quality research.

The article "Traditional Chinese Medicine Moxibustion in the Treatment of Infantile Diarrhea" was retracted in 2023. Reasons: signs of a paper mill; compromised peer review; unreliable results or conclusions.

Three researchers independently screened and extracted according to the pre-established inclusion and exclusion criteria (the researchers were all graduate students who had systematically studied evidence-based medicine courses) and checked the inclusion results. If there was a disagreement, it would be discussed or decided by the fourth researcher. The extraction content mainly includes ① Baseline level; ② Basic information of the included literature; ③ Quality of included studies; ④ The source and number of cases included; ⑤ Intervention measures; ⑥ Measurement index; ⑦ Outcome indicators.

### 2.4. Statistical Method

For the statistical analysis, we have utilized the Rev Man 5.3 software which is extremely useful for the problem at hand. A heterogeneity test was conducted for the included studies, and the degree of heterogeneity was observed according to *I*^2^ value. If *P* > 0.1, *I*^2^ < 50%, it was considered that there was homogeneity among the studies, and the fixed effect model was used; If *P* < 0.1, when *I*^2^ ≥ 50%, the random effects model was used when consistency was considered among studies and merging was needed; if *P* < 0.1, and *I*^2^ ≥ 50% and the source of heterogeneity could not be determined. Meta-analysis was not performed and descriptive analysis was used.

## 3. Results

In this section, we are going to describe in detail that what is the output of the proposed scheme when applied to the actual data? In addition, the results of the proposed study are thoroughly evaluated and are presented in both tabular and textual form. For simplicity, these are divided into numerous subsections which are given below.

### 3.1. Basic Characteristics of the Included Literature and Method Quality Assessment

A total of 215 related pieces of literature were retrieved. 138 pieces of literature were repeatedly published and obviously did not meet the inclusion criteria were excluded, and 73 pieces of literature were preliminarily screened. After reading the titles and abstracts, 29 well-designed studies were selected. Through searching the full text, reading literature, and quality evaluation, 17 papers were finally included. Basic characteristics of the included literature and method quality assessment were shown in Table 1.

### 3.2. Result of Meta-Analysis

Response rates were reported in all 17 studies, and subgroup analysis was performed based on whether or not other therapies were combined. 7 studies compared the effectiveness of simple moxibustion and conventional therapy in the treatment of infantile diarrhea, and the results showed statistically significant differences [OR = 4.01, 95% CI (2.03, 7.84), *P* < 0.0001]; 10 studies compared the effectiveness of moxibustion combined with other therapies and conventional therapies in the treatment of diarrhea in children, and the results showed that the difference had general meaning [OR = 4.45, 95% CI (2.83, 7.10), *P* < 0.00001]. The funnel plot (Figure 1) showed that the distribution of included studies was asymmetrical on both sides of the baseline, which could be considered as publication bias. The result of the Meta-analysis was shown in Table 2.

The article "Traditional Chinese Medicine Moxibustion in the Treatment of Infantile Diarrhea" was retracted in 2023. Reasons: signs of a paper mill; compromised peer review; unreliable results or conclusions.

Funnel plot was shown in Figure 1.

## 4. Discussion

Infantile diarrhea is a common digestive tract disease in pediatrics. It is mainly caused by a poor diet which damages the spleen and stomach, or by the invasion of the lung and stomach caused by the evil of wind and cold [24]. In the theory of Traditional Chinese medicine, children with diarrhea belong to “diarrhea,” spleen and stomach function damage, temper disorder, blood deficiency, spleen, and stomach weakness [25]. In modern medical theory, due to the children's younger age, immature spleen and stomach function, the digestive ability is limited, digestive enzyme secretion is insufficient, and digestive system disorders, forming a vicious circle [26]. Traditional Chinese medicine moxibustion is made of moxa stick or moxa stick with moxa as the main material. After lighting, the moxa stick is smoked and ironed or warmed to burn the body surface acupoints. By stimulating the activity of Qi to adjust the body's disordered physiological and biochemical functions, so as to achieve the purpose of disease prevention and treatment of a treatment method [27]. Traditional Chinese moxibustion has the function of warming the middle and dispersing cold, strengthening the spleen and strengthening the kidney, reducing dampness and stopping diarrhea, improving the immunity of the body, and improving the weak constitution [28]. Traditional Chinese medicine moxibustion can stimulate Qi and adjust the disorder of physiological function, before moxibustion, the symptoms of children are differentiated to determine the specific syndrome type, implementing symptomatic treatment, by selecting appropriate acupoints and stimulating acupoints, to make the digestive function of children return to normal [29, 30]. In recent years, the clinical treatment effect of Traditional Chinese moxibustion on diarrhea has become a hot research topic, especially since 2011, the research process has been rapidly accelerated [31]. Comparative analysis of the clinical efficacy of moxibustion and its comprehensive therapy on different types of diarrhea found that Traditional Chinese moxibustion for children with diarrhea treatment effect is better, can effectively shorten the course of the disease's quick recovery, reduce the inconvenience of children's intake of drugs, and significantly alleviate the symptoms of diarrhea in children [32].

The article "Traditional Chinese Medicine Moxibustion in the Treatment of Infantile Diarrhea" was retracted in 2023. Reasons: signs of a paper mill; compromised peer review; unreliable results or conclusions.

## 5. Conclusion

In this study, we have carefully read the titles and abstracts of approximately twenty-nine articles, which are available in the literature. However, the selection of these articles is based on a dedicated mechanism, i.e., inclusion and exclusion criteria, which are described in the proposed section. In the next step, we have searched the full text, reading literature, and quality evaluation through which we were able to select seventeen papers. Response rates were reported in all 17 studies, and subgroup analysis was performed based on whether or not other therapies were combined. 7 studies compared the effectiveness of simple moxibustion and conventional therapy in the treatment of infantile diarrhea, and the results showed statistically significant differences [OR = 4.01, 95% CI (2.03, 7.84), *P* < 0.0001]; 10 studies compared the effectiveness of moxibustion combined with other therapies and conventional therapies in the treatment of diarrhea in children, and the results showed that the difference had general meaning [OR = 4.45, 95% CI (2.83, 7.10), *P* < 0.00001]. The funnel plot (Figure 1) showed that the distribution of included studies was asymmetrical on both sides of the baseline, which could be considered as publication bias.

Finally, Traditional Chinese medicine moxibustion could effectively relieve the symptoms of infantile diarrhea and the effect was significant as we have observed through experiments.

## Figures and Tables

**Figure 1:** Funnel plot.

**Table 1:** Basic characteristics of the included literature and method quality-02 assessment.

Literature	Cases		Interventions		Outcome indicators	Experimental group	Control group
	Experimental group	Control group	Period of treatment	Acupuncture point			
Xu [7]	30	30	Moxibustion	Montmorillonite powder	20 min/time, 14d	Shenque	①
Xu et al. [8]	75	75	Spleen-tonifying qi powder + cistanche moxibustion	Symptomatic treatment	15 min/time, 12d	Shenque, Tianshu	②
Fang et al. [9]	43	43	Ziwuliuzhu acupoint moxibustion	Conventional treatment	4d	Shenque	②⑤
Zhai et al. [10]	38	38	Moxibustion + western medicine	Conventional western medicine	10 min/time, 10d	Shenque	①②
Huang et al. [11]	104	105	Ginger aconite cake + moxibustion	Conventional treatment	15 min/time, 7d	Qihai, Tianshu	②⑥
Jiang [12]	55	55	Moxibustion + western medicine	Conventional western medicine	15 min/time, 7d	Shenque, Zusanli	①
Meng and Zhitao [13]	39	39	Moxibustion + Western medicine	Conventional western medicine	20 min/time, 7d	Shenque	③④⑥
Zhong [14]	50	50	Moxibustion	Conventional treatment	30 min/time, 11d	Shenque, Guanyuan	②⑤⑥
Dai et al. [15]	26	26	Moxibustion + Western medicine	Conventional western medicine	10 min/time, 9d	Shenque	①⑤⑦
Cui et al. [16]	50	50	Moxibustion	Conventional treatment	25 min/time, 11d	Zhong wan,Shenque, Qihai, Guanyuan	①②
Chen et al. [17]	50	50	Moxibustion	Paste	30 min/time, 10d	Fengchi, Shenque	①
Li and Gai [18]	28	28	Moxibustion	Paste	15 min/time, 10d	Shenque	①⑤⑥ ⑦
Zhang [19]	70	70	Moxibustion	Antidiarrheal stick	30 min/time, 7d	Shenque, Qihai, Guanyuan	①
Liu [20]	55	55	Moxibustion	Conventional treatment	25 min/time,10d	Piyu	①③④
Zhang [21]	30	30	Moxibustion + massage	Conventional treatment	30 min/time, 9d	Shenque	②③④
Hu [22]	81	81	Ziwuliu moxibustion + antidiarrheal ointment	Conventional treatment	25 min/time, 10d	Shenque, Zhongwan	①②
Zhu [23]	42	42	Moxibustion + western medicine	Paste	30 min/time, 10d	Shenque, Tianshu	①②⑤

Note: the equilibria between groups were *P* > 0.05. Outcome indicators:① total effective rate; ②TCM syndrome scores; ③ the improvement time of stool; ④ abdominal pain relief time; ⑤ the time needed to reduce fever; ⑥ treatment time; ⑦ relief time of vomiting; ⑧ diarrhea relief time.

The article "Traditional Chinese Medicine Moxibustion in the Treatment of Infantile Diarrhea" was retracted in 2023. Reasons: signs of a paper mill; compromised peer review; unreliable results or conclusions.

**Table 2:** Result of Meta-analysis.

Literature	Random method	Blind method	Allocation concealment	Baseline similarity	Exit/lost
Xu Meifang	Random	Without mention	Without mention	Consistent	Without mention
Xu Zao Lin et al.	Random	Mention	Without mention	Consistent	Without mention
Fang Lina	Random	Without mention	Sequence of admission	Consistent	Without mention
Zhai Hongmin	Computer extraction	Without mention	Without mention	Consistent	Without mention
Huang Rixiang et al.	Random	Without mention	Without mention	Consistent	Without mention
Jiang Yuanyuan	Random	Without mention	Sequence of visits	Consistent	Without mention
Meng Lixian	Random	Without mention	Without mention	Consistent	Without mention
Zhong Ling	Random number table	Without mention	Without mention	Consistent	Without mention
Dai Juan et al.	Method of lottery	Without mention	Sequence of admission	Consistent	Mention
Wei Cui et al.	Random number table	Without mention	Without mention	Consistent	Without mention
Chen Yanxia et al.	Random	Without mention	Without mention	Consistent	Without mention
Li Meng et al.	Random number table	Without mention	Without mention	Consistent	Without mention
Zhang Zhaoguo	Random	Without mention	Without mention	Consistent	Mention
Liu Xingxiang	Random	Without mention	Sequence of visits	Consistent	Without mention
Zhang Liqiao	Random number table	Mention	Without mention	Consistent	Without mention
Hu Daiping	Random	Without mention	Without mention	Consistent	Without mention
Zhu Qunlei	Random	Without mention	Without mention	Consistent	Without mention

The article "Traditional Chinese Medicine Moxibustion in the Treatment of Infantile Diarrhea" was retracted in 2023. Reasons: signs of a paper mill; compromised peer review; unreliable results or conclusions.

## Data Availability

The datasets used during the present study are available from the author upon request.
